The article "Clinicopathological characteristics and prognosis of early-stage HER2 low-expression breast cancer: A single-center retrospective study" was published in 2023. Journal: Front Oncol.

# Clinicopathological characteristics and prognosis of early-stage HER2 low-expression breast cancer: A single-center retrospective study

**DOI:** 10.3389/fonc.2023.1130734

**Published:** 2023-03-29

**Authors:** Chang-Gen Liu, Yi-Fan Li, Tian-Yi Ma, Meng Lv, Zhi-Dong Lv, Yuan-Yuan Wang, Xiang-Ping Liu, Yan Mao, Hai-Bo Wang

**Affiliations:** ^1^ Breast Center, The Affiliated Hospital of Qingdao University, Qingdao, China; ^2^ Department of Medicine, Qingdao University, Qingdao, China

**Keywords:** breast cancer, HER2-low, survival, prognosis, clinicopathological features

## Abstract

**Background:**

Owing to the emergence of drugs targeting human epidermal growth factor receptor 2 (HER2), remarkable prognostic enhancement has been seen for patients with HER2-positive breast carcinoma. However, anti-HER2 medicines are applicable merely to individuals with HER2-positive tumors, and the benefit for those with low HER2 expression is unclear. The DESTINY-Breast04 phase III and RC48 clinical trial results showed the benefit of antibody-drug couples for low HER2-expressing individuals with breast carcinoma, challenging the traditional dichotomy between HER2-negative and -positive tumors. Hence, the purposes of the present work are to explore the clinicopathological traits and prognostic differences in the HER2-low expression Chinese population with early-stage breast carcinoma.

**Methods:**

Data from the database of the Breast Center of the Affiliated Hospital of Qingdao University were collected from January 2008 to December 2017. We screened a total of 4,598 patients, of which 2,837 had HER2-0 tumors and 1,761 had HER2-low tumors. Additionally, clinicopathological characteristics, survival, and prognostic information were obtained. Difference comparisons were made between HER2-0 and HER2-low groups regarding the clinical traits and outcomes.

**Results:**

We enrolled 4598 patients, with the HR-positive subjects suffering from HER2-low breast carcinoma higher in proportion than the HR-negative patients. In contrast to HER2-0 tumors, the HER2-low tumors were linked to an older median age at diagnosis, T1 tumors, N1 stage, a higher Ki-67 index, as well as inferior histological grade. Insignificant inter-group difference was noted regarding overall survival (OS), although the HER2–0 group exhibited better disease-free survival (DFS) than the HER2-low group for the entire (P = 0.003), lymph node-negative (P = 0.009) and HR-positive (P = 0.007) populations. According to the multivariate regression finding, low HER2 expression was an inferior DFS prognostic factor in the HER2-negative population with early-stage breast cancer (HR,1.33;95% CI, 1.06-1.66; P = 0.013).

The article "Clinicopathological characteristics and prognosis of early-stage HER2 low-expression breast cancer: A single-center retrospective study" was published in 2023. Journal: Front Oncol.

**Conclusion:**

The clinical traits of the HER2-low carcinomas differed from those of HER2–0 tumors. Despite the insignificant inter-group difference in OS, the differences in DFS were found for the overall, lymph node-negative and HR-positive subjects, suggesting the possibility of HER2-low as an inferior prognostic factor for disease progression in early-stage breast cancer.

## Introduction

About 15–20% of breast carcinoma sufferers express human epidermal growth factor receptor 2 (HER2) excessively, and HER2 overexpression without treatment is linked to a worse outcome (1). Owing to the advent of patuximab and trastuzumab, there has been immense outcome enhancement among the HER2-positive breast carcinoma patients (2). However, 40–50% of them express low HER2, whose ISH score was negative but IHC score 1+ or 2+ (3, 4). Most previous studies showed that targeted therapy with conventional anti-HER2 agents is inefficient for non-amplified tumors that express low/moderate levels of HER2 (5). However, recent clinical trial results suggested that novel antibody-drug couples (ADCs) potentially target HER2-low tumors. Compared with trastuzumab emtansine (T-DM1), these novel ADCs are more efficacious in killing bystanders through cleavable junction utilization, which also show higher drug/antibody ratios active in HER2-overexpressing and low-expressing tumors (6). The latest DESTINY-Breast04 phase III study showed encouraging results in 52.3% of patients in the trastuzumab deruxtecan group with objective remission and a 23.4-month median overall survival (OS) among the HER2-low metastatic breast carcinoma patients who had priorly underwent first- or second-line chemotherapy (7).

Therefore, as a novel clinical subtype, HER2-low breast carcinoma should be explored further, and its case characteristics and prognostic differences should also be investigated. Several studies showed inconsistent findings on the outcome comparison between the HER2-0 (HER2-IHC 0) and HER2-low breast carcinomas (8–10), and further studies are needed because studies in the Chinese population are still scarce. Hence, Chinese individuals having HER2-0 and HER2-low breast carcinomas were retrospectively assessed herein.

## Patients and methods

**Figure 1** outlines the process of selecting patients in the retrospective single-center research. The entire newly-diagnosed female early-stage breast carcinoma patients with negative HER2 expression, who received treatment at our center from January of 2008 to December of 2017, were enrolled. Exclusion criteria were breast carcinoma patients at stage IV, with positive HER2 expression, insufficient HER2 data, as well as lobular or ductal carcinoma in situ. We gathered the clinicopathological information from the breast carcinoma database of Qingdao University Hospital, which encompassed demographics, tumor dimensions, state of lymph nodes, HER2 level, ER and PR staining, histological grading, as well as Ki-67. A total of 4,598 patients were enrolled eventually into the analysis. We also gathered long-term outcomes in terms of survival and relapse, where the median follow-up duration was 71 months (varying from 2 to 177 months).

The article "Clinicopathological characteristics and prognosis of early-stage HER2 low-expression breast cancer: A single-center retrospective study" was published in 2023. Journal: Front Oncol.

**Figure 1:** Patients Screening Flow Chart.

In accordance with the guidelines by American Society of Clinical Oncology (ASCO)/College of American Pathologists (CAP), the HER2 status based on IHC was divided into three categories: patients were deemed to have negative, ambiguous and positive HER2 expressions when their IHC scores were 0 or 1+, 2+, and 3+, respectively. For the HER2-ambiguous subjects, their HER2 status was further examined through *in situ* hybridization (ISH). Subsequently, the ISH-positive tumors were identified as HER2-positive, while the ISH-negative tumors were recognized as HER2-negative (11). Any patient scoring 1+ or 2+ on IHC but negative on ISH were considered to express HER2 lowly (4).

HER2 testing, January 2007 to September 2013, was determined according to the 2007 edition of the ASCO/CAP guidelines, as follows:a positive HER2 result is IHC staining of 3+ (uniform, intense membrane staining of > 30% of invasive tumor cells), a fluorescent *in situ* hybridization (FISH) result of more than six HER2 gene copies per nucleus or a FISH ratio (HER2 gene signals to chromosome 17 signals) of more than 2. A negative result is an IHC staining of 0 or 1+, a FISH result of less than 4.0 HER2 gene copies per nucleus, or FISH ratio of less than 1.8. Equivocal results require additional action for final determination (12). HER2 testing determinations from October 2013 to December 2017 were based on the 2013 edition of the ASCO/CAP guidelines.Testing criteria define HER2-positive status when (on observing within an area of tumor that amounts to > 10% of contiguous and homogeneous tumor cells) there is evidence of protein overexpression (IHC) or gene amplification (HER2 copy number or HER2/CEP17 ratio by ISH based on counting at least 20 cells within the area). If results are equivocal (revised criteria), reflex testing should be performed using an alternative assay (IHC or ISH) (13).

We used 14% as the Ki-67 cut-off value based on the consensus of the 2011 St. Gallen meeting (14).

### Statistical analysis

Differences in the categorical data frequencies between HER2-low and HER2-0 groups were examined *via* χ2 or Fisher exact test. Moreover, normally-distributed continuous variables and non-normal variables were compared separately through t and Mann–Whitney tests. Survival graphs were computed by Kaplan–Meier (KM) technique, while difference comparison was accomplished *via* log-rank test. Cox regression was exploited to conduct univariate and multivariate assessments, followed by estimation of adjusted hazard ratios (HRs) plus 95% confidence intervals (CIs).

The article "Clinicopathological characteristics and prognosis of early-stage HER2 low-expression breast cancer: A single-center retrospective study" was published in 2023. Journal: Front Oncol.

The entire data were processed with the aid of SPSS ver. 22 (Chicago, IL, USA), and differences were regarded as significant when P <0.05.

Disease-free survival (DFS) referred to the duration between the date of surgery and the date of relapse or death due to any factor. Besides, OS referred to the duration between the operative date and the date of death due to any factor.

## Results

### Baseline patient characteristics

We screened 4598 patients, including 2837 HER2-0 (61.7%) and 1761 HER2-low patients (38.2%). Of the 1761 patients with HER2-low tumors, 1487 (32.3%) and 274 (5.9%) were HER2 IHC 1+ and HER2 IHC 2+, respectively. Regarding HR status, there were 3633 HR-positive (79.0%) and 965 triple-negative breast cancer (TNBC) (21.0%) patients. The baseline pathological and clinical traits are detailed in **Table 1**, which are based on the status of HER2 expression. The HR-positive subjects exhibited a higher proportion of HER2-low breast carcinoma compared to the TNBC subjects, with 1,425 (39.2%) vs. 336 (34.8.%) (P <0.05). HER2-low carcinomas were diagnosed more frequently among individuals older than 50 years in contrast to the HER2–0 carcinomas (61.8% vs. 54.4%, P <0.001), and at an older median age (53 years vs. 51 years, P <0.001). The HER2-0 group included a larger number of premenopausal patients (P <0.001). There was no difference in pathological stage (stage 1 to 3) between the two groups(P=0.188). More T1 tumors were noted in the HER2-low group, while more T2 tumors were found in the HER2-0 group (P = 0.025). Additionally, more N1 tumors were observed among the HER2-low subjects in contrast to the HER2-0 ones (25.0% vs. 21.9%, P = 0.041). The histological grading of HER2-0 carcinomas was lower than that of HER2-low carcinomas (P < 0.001). Regarding the pathological type, the HER2-low subjects exhibited higher proportion of IDC(Invasive ductal cancer) compared to the HER2-0 subjects (90.1% vs. 84.6%, P <0.001). Moreover, the proportion of patients with a Ki-67 labeling index of >14% in the HER2-low group was higher than in the HER2-IHC 0 group (73.9% vs. 65.3%, P < 0.001).

**Table 1:** Clinicopathological characteristics of patients with HER2-low breast cancer.

Variables	All patients(n=4598)	HER2-0 (n=2837)	HER2-low (n=1761)	P value*
Age,median(range)	51(20-96)	51(20-96)	53(20-95)	**0.001**
Age				**0.001**
<50	1965(42.7%)	1293(45.6%)	672(38.2%)	
≥50	2633(57.3%)	1544(54.4%)	1089(61.8%)	
Menopausal status				**0.001**
Premenopause	1752(38.1%)	1177(41.5%)	575(32.7%)	
Postmenopause	2846(61.9%)	1660(58.5%)	1186(67.3%)	
HR				**0.012**
HR-positive	3633(79.0%)	2208(77.8%)	1425(80.9%)	
HR-negative	965(21.0%)	629(22.2%)	336(19.1%)	
Pathological stage				0.188
Stage I	1728(37.6%)	1037(36.6%)	691(39.2%)	
Stage II	2235(48.6%)	1401(49.4%)	834(47.4%)	
Stage III	635(13.8%)	399(14.1%)	236(13.4%)	
T				**0.025**
≤2cm	2421(52.7%)	1451(51.1%)	970(55.1%)	
2cm-5cm	2076(45.2%)	1318(46.5%)	758(43.0%)	
>5cm	101(2.2%)	68(2.4%)	33(1.9%)	
N				**0.041**
N0	2927(63.7%)	1833(64.6%)	1094(62.1%)	
N1	1060(23.1%)	620(21.9%)	440(25.0%)	
N2	392(8.5%)	255(9.0%)	137(7.8%)	
N3	219(4.8%)	129(4.5%)	90(5.1%)	
HG				**0.001**
1	560(12.1%)	428(15.0%)	132(7.4%)	
2	2703(58.7%)	1603(56.5%)	1100(62.4%)	
3	1238(26.9%)	750(26.4%)	488(27.7%)	
Unknown	97(2.1%)	56(1.9%)	41(2.3%)	
Histological type				**0.001**
IDC	3987(86.7%)	2401(84.6%)	1586(90.1%)	
ILC	159(3.5%)	108(3.8%)	51(2.9%)	
other	452(9.8%)	328(11.6%)	124(7.0%)	
Ki-67				**0.001**
≤14%	1447(31.4%)	985(34.7%)	460(26.1%)	
>14%	3151(68.6%)	1852(65.3%)	1301(73.9%)	
Breast surgery				**0.046**
TM	3477(75.6%)	2179(76.8%)	1298(73.7%)	
BCS	876(19.1%)	519(18.3%)	357(20.3%)	
BRS	245(5.3%)	139(4.9%)	106(6.0%)	
Endocrine therapy				**0.017**
Yes	3589(78.1%)	2182(76.9%)	1407(79.9%)	
No	1009(21.9%)	655(23.1%)	354(20.1%)	
Adjuvant RT				0.263
Yes	1891(41.1%)	1150(40.5%)	741(42.1%)	
No	2235(48.6%)	1405(49.5%)	830(47.1%)	
Unknown	472(10.3%)	282(9.9%)	190(10.8%)	
CT				0.077
Adjuvant CT	3308(71.9%)	2066(72.8%)	1242(70.5%)	
Neoadjuvant CT	154(3.3%)	83(2.9%)	71(4.0%)	
No	1014(22.1%)	608(21.4%)	406(23.1%)	
Unknown	122(2.7%)	80(2.8%)	42(2.4%)	

HR,Hormone receptor; T, Tumor length diameter; N, Lymph node stage; HG, Histological grade; IDC, Invasive ductal cancer; ILC, Invasive lobular cancer; TM, Total mastectomy; BCS, Breast conserving surgery; BRS, Breast reconstruction surgery; RT, radiotherapy; CT, Chemotherapy.

The article "Clinicopathological characteristics and prognosis of early-stage HER2 low-expression breast cancer: A single-center retrospective study" was published in 2023. Journal: Front Oncol.

*Bold values indicate statistically significant results.

In terms of surgical modality, a slightly higher percentage of total mastectomies were performed in the HER2-0 group(76.8% vs. 73.7%, P=0.046).No significant differences were seen between the two groups in terms of adjuvant radiotherapy (P=0.263) and chemotherapy (P=0.077), and the HER2-low group received a higher proportion of endocrine therapy due to a higher proportion of HR-positive people(P=0.017).Chemotherapy regimens containing anthracyclines and selective estrogen receptor modulators are the most commonly used adjuvant chemotherapy and endocrine therapy regimens, respectively.

### Survival outcomes

The median follow-up time was 71 months (range, 2–177 months). During the follow-up period, 146 all-cause deaths occurred. As revealed by the KM survival graphs, the OS of HER2-0 group differed insignificantly from that of HER2-low group, regardless of the HR and lymph nodestatus (**Figures 2A–E**). However, the DFS for HER2–0 subjects was superior to that for HER2-low subjects in the overall enrolled population, separately showing five-year rates of DFS of 94.3% and 92.7% (P = 0.003; **Figure 3A**). Additionally, similar results were seen in the HR-positive breast cancer population, with a five-year DFS being 94.8% for the HER2-0 subjects and 93.6% for the HER2-low subjects (P = 0.007; **Figure 3B**). Conversely, the DFS difference between these 2 groups was insignificant for the HR-negative breast cancer population(P = 0.089; **Figure 3C**).Exploratory subgroup analysis based on lymph node status showed superior DFS among HER2–0 subjects to the HER2-low subjects for the lymph node-negative population (96.3% vs. 94.7%, P = 0.009; **Figure 3D**), whereas for the lymph node-positive population, an insignificant 5-year DFS difference was noted between the HER2-0 and HER2-low subjects (90.6% vs. 89.5%, P = 0.196; **Figure 3E**).

**Figure 2:** Kaplan–Meier survival curves for OS stratified by hormone receptor (HR) status and lymph node status.OS for HER2-low vs. HER2-0 tumors in the complete cohort **(A)**, HR-positive population **(B)**, HR-negative population **(C)**, Lymph node-negative population **(D)** and lymph node-positive population **(E)**. p values are from the stratified log-rank test.

**Figure 3:** Kaplan–Meier survival curves for DFS stratified by hormone receptor (HR) status and lymph node status.DFS for HER2-low vs. HER2-0 tumors in the complete cohort **(A)**, HR-positive population **(B)**, HR-negative population **(C)**, Lymph node-negative population **(D)** and lymph node-positive population **(E)**. p values are from the stratified log-rank test.

The **Tables 2**–**4** shows the univariate and multivariate analyses of DFS clinicopathological factors. According to the univariate findings, tumor size, lymph node stage, hormone receptor negativity, high histologic grade, high Ki-67 and low HER2 level were linked to inferior DFS for the entire included patients. In multivariate analysis, tumor size, lymph node stage, hormone receptor negativity, high histologic grade, high Ki-67 and low HER2 level were linked to inferior DFS for the entire enrolled patients (**Table 2**). COX analysis showed similar results among the HR-positive population (**Table 3**). But in the lymph node-negative population, postmenopause, tumor size, and high histologic grade were not statistically associated with poorer DFS in the univariate analysis, and hormone receptor negativity, high Ki-67 and low HER2 level were linked to poorer DFS. In multifactorial analysis, correlations of hormone receptor negativity, high Ki-67, as well as low HER2 level with poorer DFS were noted among the lymph node-negative population (**Table 4**).

The article "Clinicopathological characteristics and prognosis of early-stage HER2 low-expression breast cancer: A single-center retrospective study" was published in 2023. Journal: Front Oncol.

**Table 2:** Univariate and multivariate analyses for disease-free survival in the overall population.

Variables	Multivariate analysis HR(95%Cl)	P value*	Univariate annalysis HR(95%Cl)	P value*
T				
≤2cm	1.00			
2cm-5cm	1.76(1.41-2.21)	**0.001**	1.43(1.14-1.80)	**0.002**
>5cm	4.80(3.10-7.43)	**0.001**	3.28(2.09-5.14)	**0.001**
N				
N0	1.00			
N1	1.63(1.25-2.13)	**0.001**	1.56(1.19-2.04)	**0.001**
N2	2.93(2.16-3.96)	**0.001**	2.60(1.90-3.56)	**0.001**
N3	5.21(3.79-7.16)	**0.001**	4.44(3.19-6.18)	**0.001**
Hormone receptor-negative/ positive	1.40(1.11-1.77)	**0.005**	1.35(1.02-1.79)	**0.038**
HER2-low/HER2-0	1.39(1.12-1.73)	**0.003**	1.33(1.06-1.66)	**0.013**
Ki-67>14%/≤14%	1.60(1.25-2.06)	**0.001**	1.31(1.01-1.69)	**0.041**
HG				
1	1.00			
2	1.87(1.22-2.85)	**0.004**	1.78(1.16-2.72)	**0.008**
3	2.31(1.49-3.59)	**0.001**	1.71(1.07-2.73)	**0.024**

HR, hazard ratio; CI, confidence interval; T, Tumor length diameter; N, Lymph node stage; HG, Histological grade.

*Bold values indicate statistically significant results.

**Table 3:** Univariate and multivariate analyses for disease-free survival in the Hormone receptor-positive population.

Variables	Multivariate analysis HR(95%Cl)	P value*	Univariate annalysis HR(95%Cl)	P value*
T				
≤2cm	1.00			
2cm-5cm	2.04(1.57-2.66)	**0.001**	1.63(1.24-2.15)	**0.001**
>5cm	5.58(3.27-9.51)	**0.001**	3.37(1.93-5.88)	**0.001**
N				
N0	1.00			
N1	1.69(1.23-2.30)	**0.001**	1.49(1.08-2.04)	**0.014**
N2	3.07(2.15-4.37)	**0.001**	2.50(1.73-3.60)	**0.001**
N3	5.59(3.86-8.09)	**0.001**	4.26(2.89-6.28)	**0.001**
HER2-low/HER2-0	1.43(1.10-1.85)	**0.007**	1.33(1.02-1.73)	**0.036**
Ki-67>14%/≤14%	1.63(1.23-2.16)	**0.001**	1.34(1.01-1.78)	**0.041**
HG				
1	1.00			
2	2.06(1.28-3.32)	**0.003**	1.95(1.21-3.15)	**0.006**
3	3.21(1.92-5.38)	**0.001**	2.66(1.58-4.47)	**0.001**

HR, hazard ratio; CI, confidence interval; T, Tumor length diameter; N, Lymph node stage; HG, Histological grade.

*Bold values indicate statistically significant results.

**Table 4:** Univariate and multivariate analyses for disease-free survival in the Lymph node-negative population.

Variables	Multivariate analysis HR(95%Cl)	P value*	Univariate annalysis HR(95%Cl)	P value*
T				
≤2cm	1.00			
2cm-5cm	1.25(0.91-1.73)	0.171	1.20(0.86-1.67)	0.281
>5cm	1.85(0.68-5.06)	0.23	1.87(0.68-5.14)	0.227
Hormone receptor-negative/ positive	1.52(1.08-2.14)	**0.016**	1.65(1.20-2.48)	**0.016**
HER2-low/HER2-0	1.55(1.11-2.16)	**0.009**	1.60(1.15-2.24)	**0.006**
Ki-67>14%/≤14%	2.05(1.39-3.02)	**0.001**	1.85(1.24-2.76)	**0.003**
HG				
1	1.00			
2	0.87(0.54-1.38)	0.546	0.73(0.45-1.17)	0.186
3	0.88(0.52-1.48)	0.624	0.52(0.29-0.93)	**0.028**

HR, hazard ratio; CI, confidence interval; T, Tumor length diameter; N, Lymph node stage; HG, Histological grade.

The article "Clinicopathological characteristics and prognosis of early-stage HER2 low-expression breast cancer: A single-center retrospective study" was published in 2023. Journal: Front Oncol.

*Bold values indicate statistically significant results.

## Discussion

Our results showed that low HER2 expression accounted for 38.2% of the HER2-negative population, which was similar to that of previous studies reporting that approximately 40–50% of breast carcinoma patients express HER2 lowly (8, 9, 15, 16). Low HER2 expression may vary by the status of HR, with the HR-positive population having a higher proportion of HER2-low breast carcinoma. Moreover, HER2-low breast cancer has different clinicopathologic characteristics from the HER2-0 one. In contrast to the HER2-0 carcinomas, the HER2-low carcinomas are diagnosed at a higher median age, more frequently occur in postmenopausal population, and are linked to more T1 tumors, higher N1 staging, worse histologic grading, and higher Ki-67 index.

In terms of survival, the OS between the HER2-low and HER2–0 groups was not significantly different irrespective of the HR status, although the HER2–0 subjects exhibited superior five-year DFS to the HER2-low subjects for the entire, lymph node-negative and HR-positive populations. Moreover, Cox regression analysis recognized low HER2 level as an independent inferior prognostic factor that is linked to DFS. The mechanism describing the adverse prognostic impact of HER2-low in early-stage breast cancer is unclear, which may be related to its worse clinicopathological factors. However, further investigation is necessary to examine its more complex biological differences. Many previous studies suggested that HER2-low breast cancer may be a clinically and biologically distinct subtype that may affect patient prognosis (17), and for early-stage breast carcinoma patients, a low HER2 level can negatively affect prognosis even without HER2 amplification (10, 18–21). The HR-positive breast carcinoma sufferers with moderate HER2-expressing HER2 2+ have been reported to exhibit inferior DFS to those with HER2 1+ or 0 but no difference in BCSS (breast carcinoma-specific survival: duration between the operative date and the date of final follow-up or breast carcinoma-induced death) (20). In another report, subjects aged 55+ years with HER2 2+ expression had a worse prognosis compared with HER2 0/1+ subjects, showing an HR of 1.45 and 95% CIs of 1.01–2.07 (P = 0.044) (21). Moderate HER2(2+) status is defined as having 500,000 detectable HER2 receptors on the cell surface, which are required to activate the essential intracellular HER2 pathway to drive tumor growth and invasion (22).In contrast, a relatively small proportion of HER2 2+ patients had a negative prognostic impact with low level of HER2, scoring 1+ or 2+ on IHC but negative on FISH, suggesting that HER2 IHC 1+ may have similar biological behavior with HER2 IHC 2+ that could adversely affect prognosis. HER2 low-expressing tumors may be more sensitive to different growth factors that stimulate breast cancer cells, as HER2 signaling is a key factor in breast cancer proliferation (22).In addition, the prognosis of lymph node-negative patients is usually better than lymph node-positive patients. However, low HER2 expression in lymph node-negative patients was also an independent poor prognostic factor for DFS, but further large-scale prospective studies should be conducted to confirm whether low HER2 expression could be used as a reference indicator for further intensive treatment in early-stage breast cancer.

The article "Clinicopathological characteristics and prognosis of early-stage HER2 low-expression breast cancer: A single-center retrospective study" was published in 2023. Journal: Front Oncol.

We revisited the HER2 low-expression population because of the recent release of phase III results from the DESTINY-Breast04 clinical trial due to the emergence of novel anti-HER2 antibody-drug couples; however, the results were inconsistent in some current studies in the HER2-low expression population. In other researches, the clinical prognosis of HER2-low breast carcinoma resembled or was superior to that of HER2-0 breast cancer (9, 23, 24). Exploiting data from 4 prospective clinical neoadjuvant trials analyzing the OS and DFS differences between HER2-0 and HER2-low breast carcinomas, Denkt et al. observed a trend toward longer OS and DFS among HER2-low subjects for the HR-positive population, without presenting statistical significance (9). Won et al. analyzed 30,491 Korean patients with stage I–III breast carcinoma, discovering an insignificant OS difference between the HER2–0 and HER2-low groups. The HER2-low breast carcinoma subjects displayed prominently superior BCSS to the HER2-0 subjects (24). In addition, the prognostic impact of HER2 varies perhaps by the stage of breast carcinoma. As indicated by an analytical research involving 1,433 metastatic breast carcinoma patients based on the database of National Cancer Center in China, the HER2-low group exhibited significantly prolonged survival compared to the HER2-0 group for the entire (48.5 months vs. 43.0 months, P = 0.004) and HR-positive (54.9 months vs. 48.1 months, P = 0.011) populations, but not for the HR-negative (29.5 months vs. 29.9 months, P = 0.718) population.Recently, a study concerning breast carcinoma from Italy characterized the dynamic evolution of low HER2 expression, finding that low HER2 expression levels were significantly different between early and advanced stages, with HER2 elevations in advanced stages (25). Therefore, further research is required to explore the differences in how the low HER2 level influences treatment response and prognosis.Our findings provide evidence that HER2 low expression is biologically distinct from HER2 zero expression. We believe that the prognostic significance of low HER2 expression needs to be re-evaluated as a predictor of anti-HER2 therapy.

The article "Clinicopathological characteristics and prognosis of early-stage HER2 low-expression breast cancer: A single-center retrospective study" was published in 2023. Journal: Front Oncol.

Finally, patients in the present trial were included depending on the status of HER2 as defined by the ASCO/CAP guidelines, i.e. scoring 1+ or 2+ on IHC test, alongside negative ISH score. Because more ADC drug clinical trials demonstrate benefits in HER2 low-expressing tumors, further exploration on the current algorithm for HER2 diagnosis is required, so that the HER2 quantification approaches with higher reliability can be introduced to screen for a larger population of benefit.

The present study has a few shortcomings. First deficiency was the retrospective single-center design. Bias may be present because patients with no documented HER2 information and missing pathology information were excluded. Second, ER, PR, and HER2 status were assessed from the pathology reports of our center. Finally, the entire enrolled subjects were Chinese. Because of possible differences in cancer biology between races, these results should be interpreted with caution.

## Conclusions

We found that approximately 38% of patients with early-stage breast cancer showed low HER2 expression. A higher proportion of HR-positive patients expressed HER2 lowly compared to the TNBC patients. Despite insignificant OS difference between the HER2-0 and HER2-low groups, the former exhibited superior DFS to the latter in the overall, HR-positive, and lymph node-negative populations, which was further confirmed by multifactorial analysis, suggesting the possibility of HER2-low as an inferior prognostic factor of breast carcinomas at an early stage. With the implementation of clinical trials concerning HER2-low breast cancer and the maturing concept of HER-2 status, more studies suggest HER2-low as a new biological subtype. Therefore, larger studies are needed to elucidate the prognostic impact of HER2-low, as well as to explain it at the molecular level.

## Data availability statement

The raw data supporting the conclusions of this article will be made available by the authors, without undue reservation.

The article "Clinicopathological characteristics and prognosis of early-stage HER2 low-expression breast cancer: A single-center retrospective study" was published in 2023. Journal: Front Oncol.

## Ethics statement

The studies involving human participants were reviewed and approved by the ethics and research committee of the Affiliated Hospital of Qingdao University.Written informed consent for participation was not required for this study in accordance with the national legislation and the institutional requirements.

## Author contributions

C-GL: article writing, data collection and analysis. Y-FL, T-YM, ML, Z-DL,Y-YW and X-PL: data extraction. H-BW and YM: study design and supervision. All authors contributed to the article and approved the submitted version. 
